# Multimodal magnetic resonance imaging analysis in the characteristics of Wilson’s disease: A case report and literature review

**DOI:** 10.1515/biol-2021-0071

**Published:** 2021-08-16

**Authors:** Yun Wang, Zejin Jia, Yuelei Lyu, Qian Dong, Shujuan Li, Wenli Hu

**Affiliations:** Department of Neurology, Beijing Chao-Yang Hospital, Capital Medical University, No. 8 Gongtinan Road, Chaoyang District, Beijing 100020, China; Department of Imaging, Beijing Chao-Yang Hospital, Capital Medical University, No. 8 Gongtinan Road, Chaoyang District, Beijing 100020, China

**Keywords:** multimodal MRI, Wilson’s disease, copper, susceptibility-weighted imaging, arterial spin labeling

## Abstract

Wilson’s disease (WD) is an inherited disorder of copper metabolism. Multimodal magnetic resonance imaging (MRI) has been reported to provide evidence of the extent and severity of brain lesions. However, there are few studies related to the diagnosis of WD with multimodal MRI. Here, we reported a WD patient who was subjected to Sanger sequencing, conventional MRI, and multimodal MRI examinations, including susceptibility-weighted imaging (SWI) and arterial spin labeling (ASL). Sanger sequencing demonstrated two pathogenic mutations in exon 8 of the ATP7B gene. Slit-lamp examination revealed the presence of Kayser–Fleischer rings in both eyes, as well as low serum ceruloplasmin and high 24-h urinary copper excretion on admission. Although the substantia nigra, red nucleus, and lenticular nucleus on T1-weighted imaging and T2-weighted imaging were normal, SWI and ASL showed hypointensities in these regions. Besides, decreased cerebral blood flow was found in the lenticular nucleus and the head of caudate nucleus. The patient recovered well after 1 year and 9 months of follow-up, with only a Unified Wilson Disease Rating Scale score of 1 for neurological symptom. Brain multimodal MRI provided a thorough insight into the WD, which might make up for the deficiency of conventional MRI.

## 1 Introduction

Wilson’s disease (WD) is an autosomal recessive inherited disorder of copper metabolism, with a lifetime prevalence of 20–100% [1]. Adolescents and adults with WD may develop neurological and psychiatric diseases, including movement disorders (Parkinson, ataxia, and dystonia), cognitive impairment, depression, psychosis, and schizophrenia, which may be due to the different locations and concentrations of copper ions in various organs, resulting in excess copper accumulation in the brain, liver, kidneys, and cornea [2,3]. Grover et al. have found that a young WD patient developed psychotic symptoms characterized by irritability, delusion of persecution, and decreased sleep [1]. WD is potentially curable, suggesting immediate diagnostic evaluation and early treatment initiation of the disease [4].

Brain magnetic resonance imaging (MRI) is a crucial tool that can provide evidence of the morphological characteristics and functional changes of brain lesions, and abnormalities in brain MRI are present in more than 90% of neurological WD patients [5]. Multimodal MRI techniques, such as susceptibility-weighted imaging (SWI), arterial spin labeling (ASL), magnetic resonance spectroscopy (MRS), resting-state functional MRI, and diffusion tensor imaging (DTI), have been widely used for the clinical diagnosis of cancers, cerebral infarction, and neural degenerative diseases [6–8]. The MRI features of untreated WD cases are central pontine myelinolysis-like abnormality, tectal plate hyperintensity, giant panda face, and synchronous signal changes in thalamus, brain stem, and basal ganglia [9]. Previous research has pointed out that the damage to thalamus in WD patients can be detected using DTI prior to the abnormal signals on conventional MRI [10,11]. However, the applications of multimodal MRI in WD are rarely studied.

In this report, we described the case of a 26-year-old WD man who underwent brain multimodal MRI and reviewed the relevant literature with respect to multimodal MRI in WD patients.

## 2 Case presentation

A 26-year-old man, presented to the hospital with a mood of gloom and wretchedness, has been diagnosed with depression and treated with antidepressants. It should be noted that this patient had no history of liver disease or mental illness. After 1 month, the patient developed slow movement, slurred speech, and hand tremors, and even occasionally felt irritable. After 4 months, he was re-admitted to the hospital due to stiffness of extremities that caused difficulty in ambulation and tremors, with worsening slurred speech. On admission, the neurological examination revealed that the patient had difficulty in speaking, slight weakness (left lower limb), increased muscle tone (trunk and extremities), tremors (head and extremities), limb ataxia (left), hypoalgesia (left lower limb), and positive Babinski sign (left). Slit-lamp examination showed the presence of Kayser–Fleischer (K–F) rings in both eyes (zigzag score: 2) (Figure 1). Besides, his serum ceruloplasmin was 4.6 mg/dL and the 24-h urinary copper excretion was 204 μg/24 h. The blood cell count, serum aspartate aminotransferase level, alanine aminotransferase level, and creatinine of the patient were all normal.

**Figure 1:** K–F rings in the patient (left eye).

Subsequently, the patient was subjected to genetic test. Sanger sequencing revealed two heterozygous mutations in exon 8 of ATP7B gene, namely c.2333G>T (Arg778Leu) and c.2294A>G (Asp765Gly), of which the former mutation was inherited from his mother and the latter was from his father. Overall, the patient was diagnosed with WD based on a Leipzig score of 12, with 2 scores for K–F rings, 2 scores for ceruloplasmin, 2 scores for severe neuropsychiatric symptoms, and 4 scores for disease-causing mutation (two chromosomes). Moreover, he was examined using the Unified Wilson Disease Rating Scale (UWDRS), and the results showed that his total score was 110 on admission, including neurological score of 91, psychiatric score of 19, and liver score of 0.

MRI observations of the WD case were recorded via MRI semiquantitative scale. Brain MRI showed abnormal findings and was characterized by evidence of atrophy and signal intensity changes, with a high MRI score of 11 (Table 1). The assessment of T2-weighted imaging-fluid attenuated inversion recovery (T2WI-FLAIR)/SWI signal intensity changes was performed subjectively, while the degree of atrophy was visually assessed based on the sulcal and ventricular enlargement. Conventional brain MRI (General Electric Company, USA) results showed symmetrical hyperintensity in the midbrain and cerebral peduncle and hypointensity in the substantia nigra and red nucleus on T2WI-FLAIR (Figure 2a–c), hyperintense in the pons on T2WI-FLAIR (Figure 2d), and hypointensity in the midbrain on T1-weighted imaging (T1WI) (Figure 2e). SWI showed marked hypointensity in the substantia nigra, red nucleus, and lenticular nucleus (Figure 3a and b). ASL-MRI showed a slight decrease in cerebral blood flow (CBF) to the lenticular nucleus, with the left and right putamen being 40.4 mL/100 g/min and 38.5 mL/100 g/min, respectively (Figure 3c and d). The lenticular nucleus had no obvious abnormality on T1WI and T2WI (Figure 3e and f) (Table 1). The MRS changes of the patient in the lenticular nucleus and midbrain were unremarkable. A contrast-enhanced MRI of the abdomen revealed splenomegaly.

**Table 1:** Brain magnetic resonance imaging severity scale for Wilson disease

Parameters		Grade
Caudate nucleus	Right	1
Putamen	SWI hypointensity	1
Internal capsule	Normal	0
Thalamus	Normal	0
Midbrain	Atrophy + T2 hyperintensity + SWI hypointensity (substantia nigra and red nucleus) and giant panda face	3
Pons	Atrophy + central pontine myelinosis-like changes	3
Medulla obligation	Atrophy	1
Cerebellum	Atrophy	1
White matter	Normal	0
Cortex	Atrophy	1
Total MRI score (0–30)	—	11

SWI: susceptibility-weighted imaging. The anatomic distribution of abnormalities was noted and severity was graded based on the changes in signal intensity of focal lesions and associated atrophy: 0 = no abnormality, 1 = change in signal intensity with no atrophy or atrophy without signal change, 2 = change in signal intensity with mild or moderate atrophy, and 3 = change in signal intensity with severe atrophy. The grading system provided a score of 0–30, with 0 being the normal scan and 30 indicating the most severe changes.

**Figure 2:** Conventional brain MRI of WD. Lesions were hyperintense in the midbrain and cerebral peduncle and hypointense in the substantial nigra and red nucleus on (a) axial and (b and c) coronal T2WI-FLAIR, (d) hyperintense in the pons on T2WI-FLAIR, and (e) hypointensity in the midbrain on axial T1WI.

**Figure 3:** SWI and ASL-MRI of WD. (a and b) SWI showed decreased signal intensities in putamen, globus pallidus, substantia nigra, and red nucleus. (c and d) ASL-MRI demonstrated the reduction of cerebral blood flow in the bilateral putamen. (e) T1WI, and (f) T2WI showed substantially normal in the putamen, globus pallidus, substantial nigra, and red nucleus.

The patient was administered intravenously with dimercaptopropane sulfonate in the hospital. After discharge, the UWDRS score of the patient was 53 consisting of neurological score of 47, psychiatric score of 6, and liver score of 0. He continued oral treatment with a combination of d-penicillamine and zinc sulfate for long-term therapy and was restricted to a copper diet. After 3 months of therapy, the symptoms of speech difficulty, tremors, and stiffening of extremities remarkably improved, but the MRI remained unchanged. After 1 year and 9 months of follow-up, except for slow speech speed and slightly unclear speech, the patient recovered well and had returned to work, with only a UWDRS score of 1 for neurological symptom.

**Informed consent:** Informed consent has been obtained from all individuals included in this study.**Ethical approval:** The research related to human use has been complied with all the relevant national regulations, institutional policies, and in accordance with the tenets of the Helsinki Declaration, and has been approved by the Ethics Committee of the Beijing Chao-Yang Hospital, Capital Medical University.

## 3 Discussion

WD is an autosomal recessive disorder of copper metabolism caused by ATP7B gene mutation [12]. According to the criterion of the European Commission on Public Health and Institute of Human Genetics, WD is considered a rare disease with a prevalence of 0.0018–0.003%, suggesting the importance of intervention for WD patients [13]. The traditional WD testing depends on the assessment of urine and liver copper levels, K–F ring, ceruloplasmin, and liver-related histological changes [9]. Likewise, K–F rings were noticed in both eyes of the patient in this study, accompanied with low serum ceruloplasmin and high urine copper level. Moreover, two heterozygous mutations in exon 8 of ATP7B gene were also found in the patient, namely c.2333G>T (Arg778Leu) and c.2294A>G (Asp765Gly). Genetic testing is also a typical diagnostic technique, whereas its clinical application is limited by high costs and a large number of mutations [14].

Studies have reported that MRI is of great significance for the clinical observation and prognosis evaluation of WD patients presenting with neurological symptoms [10]. Nevertheless, the conventional MRI had a certain omission diagnostic rate [15]. Multimodal MRI refers to the combination of conventional MR scanning sequences and multiple functional MRI techniques, thereby achieving the complementary functions of multiple scanning sequences, and provides more detailed information for the diagnosis of diseases [16]. Although multimodal MRI has not been used as a diagnostic criterion for the WD due to its late emergence, evidence indicates that it exerts higher sensitivity and specificity in the detection of WD when compared with conventional MRI [6,8]. In this study, multimodal MRI techniques, including ASL and SWI, were used to describe the characteristics of neurologic WD.

SWI takes advantage of differences in magnetic susceptibility between tissues to show deposition of paramagnetic material and is particularly sensitive to iron [17]. An increasing number of studies have pointed out a complex relationship between copper and iron metabolisms in WD [18,19]. The deletion of the coding ceruloplasmin gene can cause large amounts of iron deposition in the liver and brain [20]. Several researchers have found that the liver biopsies of WD patients after long-term decoppering therapy showed a significant reduction in copper and an increase in iron, suggesting that iron overload might be associated with aceruloplasminemia [21,22]. Yang et al. have claimed that paramagnetic mineralization deposition exists in the brain gray nuclei of WD patients, and SWI is an effective approach to assess these structures, suggesting that SWI could be used as a potential biomarker for WD diagnosis [23]. The SWI results of the case showed marked dark-signal intensities in the substantia nigra, red nucleus, and lenticular nucleus despite normal T1 and T2 signals, indicating abnormal paramagnetic substance deposition in his brain.

ASL perfusion MRI sequences can be adopted for MRI-based CBF quantification without the requirement for contrast administration [24]. Ishida et al. found diffuse cerebral perfusion reduction including basal ganglia in WD patients via single-photon emission computed tomography [25]. In addition, the association between CBF and functional connectivity strength in WD patients was significantly reduced in the basal ganglia and cerebellum and slightly increased in the prefrontal cortex and thalamus compared with healthy controls. These findings suggested that aberrant coupling between resting-state CBF and functional connectivity may be a potential neural mechanism underlying the pathophysiology of WD [26]. Furthermore, the decrease in CBF in basal ganglia may be the result of neuronal loss due to copper deposition in WD. The ASL result of the patient showed slightly decreased CBF in the lenticular nucleus and the head of the caudate nucleus.

In contrast to MRI, MRS can be used to assess the concentration of different metabolites in tissues and to monitor the neurochemistry of the brain. It has been suggested that copper-induced cell injury results in reduced N-alanine aspartate/creatine ratio in WD patients, which may be partially reversed after chelation treatment [27]. A study conducted by Alkhalik Basha et al. found that there were significant differences in the mean values of N-alanine aspartate, choline, creatine, and N-alanine aspartate/creatine in MRS between WD patients and control groups, while no abnormalities were noticed in brain MRI, indicating that MRS can assist MRI in the assessment of WD [6]. In the current research, no significant change was observed in the lenticular nucleus and midbrain of the WD patient.

At present, the main available drugs for WD treatment include zinc salts and copper chelators (d-penicillamine, trientine, dimercaptopropane sulfonate, and dimercaptosuccinic acid) [28]. As the first orally administered chelating agent, d-penicillamine is effective for WD. Both d-penicillamine and zinc sulfate are the first choice for the diagnosis and treatment of WD in China [29]. However, up to 20% of WD patients have reported paradoxical worsening of neurological symptoms in the early stage of therapy, which might be associated with d-penicillamine administration [30]. Thus, the international WD diagnostic guidelines recommend trientine for patients intolerant to d-penicillamine [31], but trientine has not been used clinically in China. In addition, dimercaptopropane sulfonate combined with zinc has been proved to be an optimal therapeutic approach for neurological WD [32]. In this research, the patient was given dimercaptopropane sulfonate intravenously during hospitalization and received long-term therapy of d-penicillamine and zinc sulfate after discharge. In China, additional dimercaptosuccinic acid is needed for WD patients with d-penicillamine allergy or intolerance. Our patient had no intolerance or allergy after taking d-penicillamine orally, so dimercaptosuccinic acid was not added.

## 4 Conclusion

In this study, substantia nigra, red nucleus, and lenticular nucleus are the most involved areas, and the signals of SWI and ASL decreased in these lesions despite T1 and T2 signals are normal, suggesting that SWI and ASL may be the most sensitive sequence for neurologic WD. This is the first article to retrospect multimodal MRI features in the diagnosis of WD, illustrating the imaging characteristics of WD and enriching our knowledge with the brain multimodal MRI results. In summary, brain multimodal MRI may make up for the shortcomings of conventional MRI, and that it is useful for the diagnosis of WD. More cases with brain multimodal MRI are required to replicate these findings.
